The article "Effects of the Training of Aerobic Function on Clinical Symptoms and Quality of Life in Patients with Medium and Advanced Lung Cancer" was retracted in 2023. Reason: concerns about the peer review.

# Effects of the Training of Aerobic Function on Clinical Symptoms and Quality of Life in Patients with Medium and Advanced Lung Cancer

**DOI:** 10.1155/2022/6753959

**Published:** 2022-03-23

**Authors:** Xiangyan Lv, Yan Zhao, Yuqin Wu

**Affiliations:** ^1^ICU, The Second Affiliated Hospital of Zhejiang Chinese Medical University, Hangzhou 310005, Zhejiang, China; ^2^Department of Neurosurgery, The Second Affiliated Hospital of Zhejiang Chinese Medical University, Hangzhou 310005, Zhejiang, China

## Abstract

**Objective:**

To investigate the effects of the training of aerobic function on clinical symptoms and quality of life in patients with medium and advanced lung cancer.

**Methods:**

The study objects were 84 patients with medium and advanced lung cancer who were treated in our hospital (July 2019–July 2021) and their materials were retrospectively reviewed. Depending on the different intervention modes, they were equally divided into control group (routine nursing intervention measures) and experiment group (training of aerobic function), with 42 cases in each group. The clinical symptoms and living quality were compared between the two groups.

**Results:**

After intervention, affective meaning, behavior/severity, cognitive/mood, and sensory scores in both groups were decreased, and the various indexes in the experiment group were lower compared with the control group (*P* < 0.05). After intervention, the patients' clinical symptoms, such as pain, inappetence, insomnia, and dyspnea in the two groups were improved, and the experiment group achieved eminently better improvement compared with the control group (*P* < 0.05). After intervention, the walking distances in 6 minute walk test (6MWT) in both groups were increased, and the experiment group achieved observably longer walking distance compared with the control group (*P* < 0.05). After intervention, the patients' pulmonary function indexes of forced vital capacity (FVC), forced expiratory volume in 1s (FEV1), and FEV1/FVC% level in the two groups were all improved, and the experiment group had signally better indexes compared with the control group (*P* < 0.05). After intervention, the patients' scores of Quality of Life Questionnaire-Core Questionnaire (QLQ-C30) in both groups were decreased, and the experiment group achieved much lower score compared with the control group (*P* < 0.05).

**Conclusion:**

The training of aerobic function has obvious therapeutic effect on medium and advanced lung cancer. This training can mitigate the patients' cancer-related fatigue and clinical symptoms, improve their pulmonary function, and enhance their athletic ability and quality of life.

## 1. Introduction

Lung cancer, as one of the most common primary malignant tumors occurred in lung, originates from the bronchial epithelium or glands in the lung [1]. The early symptoms of the patients with lung cancer are not obvious, so most patients have already suffered from medium and advanced lung cancer when they are diagnosed, and they have such associated symptoms as cough, bloody sputum or hemoptysis, dyspnea, and chest pain, which seriously threaten their physical health and life safety. The etiology of lung cancer is still not completely clear at present, and a large amount of data indicate that its pathogenic factors mainly include smoking, occupational exposure, air pollution, ionizing radiation, dietary habit, genetics, history of lung diseases, and so on. For the patients with medium and advanced lung cancer, the radiochemotherapy is an indispensable treatment, but it tends to cause nausea, vomiting, pain, fatigue, reduced physical activity endurance and other adverse symptoms, and affect the patients' respiratory system, resulting in the deterioration of their quality of life [2, 3]. Therefore, effective nursing and rehabilitation training, along with the treatment, are needed to be given to the patients to relieve their clinical symptoms and improve their quality of life. Related studies [4, 5] have shown that the training of aerobic function can enhance the pulmonary function and athletic ability and has obvious therapeutic effect on chronic obstructive pulmonary diseases and cerebral infarction. According to a study of the patients with heart failure [6], the training of aerobic function shows evident effect on relieving the patients' clinical symptoms and improving their prognostic living quality. From the theoretical perspective, the training of aerobic function serves as a kind of long-distance endurance training. This training, through the continuous and repeated activities as well as the dynamic exercise lasting for some time, enhances the body's oxidative metabolism and improves the patient's cardiopulmonary function and exercise endurance, speeding up their recovery [7–9]. Based on this, the author believes that the training of aerobic function is expected to improve the patients' clinical symptoms and quality of life. However, there are few relevant studies and research data for reference in clinical practice. Hence, in this paper, the materials of 84 cases with medium and advanced lung cancer treated in our hospital were retrospectively reviewed, and the effects of the training of aerobic function on clinical symptoms and quality of life in these patients were analyzed.

## 2. Materials and Methods

### 2.1. Screening and Grouping

The study objects included 84 patients with medium and advanced lung cancer who were treated in our hospital (July 2019–July 2021) and their materials were retrospectively reviewed. Depending on the different intervention modes, they were equally divided into the control group (routine nursing intervention measures) and the experiment group (training of aerobic function), with 42 cases in each group. This study conformed with the Declaration of Helsinki [10].

### 2.2. Inclusion and Exclusion Criteria

Inclusion criteria are as follows: (1) The patients met the diagnostic criteria for medium and advanced lung cancer in Chinese Medical Association Guidelines for Clinical Diagnosis and Treatment of Lung Cancer (2018 edition) [11] and were diagnosed as lung cancer by pathological and imaging examination. (2) The patients possessed cognitive and communication ability. (3) The patients' expected survival time exceeded 6 months and their physical conditions could support them to conduct the 6-month intervention of aerobic exercise. (4) The patients and their families were informed of this study and had signed the informed consent.

Exclusion criteria are as follows: (1) The patients were complicated with severe liver dysfunction and renal dysfunction. (2) The patients suffered from coagulation disorders. (3) The patients suffered from mental illness. (4) The patients were complicated with hypertension, heart disease, and other somatic diseases.

### 2.3. Methods

The control group received routine nursing intervention measures. The nursing staff understood and analyzed the patients' basic conditions in detail and offered them knowledge education. The patients were informed of relevant knowledge of the disease, including the etiological factors, matters needing attention, and adverse symptoms. The nursing staff introduced the specific procedures and methods of treatment and nursing to patients, helped them to make mental preparation, and offered them mental nursing. Besides, the nursing staff promoted communication with the patients to understand their psychological states and offered psychological counseling to ease their negative emotions according to the actual conditions. The patients were guided to have a reasonable diet, to cultivate good living habits, to quit smoking and drinking, and to follow the doctor's advice on medication. The patients received exercise instructions based on their actual conditions.

The experiment group received the training of aerobic function on the basis of routine nursing intervention measures. The specific contents were as follows: (1) Health publicity and education: the patients were informed of the importance of implementing the training of aerobic function during treatment, and of the methods, requirements and matters needing attention of the training. (2) Formulation of exercise programs: according to the aerobic exercise prescription as well as the patients' disease statuses, ages, and physical conditions, the suitable exercise programs were formulated for them, and they were required to strictly perform the exercise programs. (3) Exercise modes: the appropriate exercises were chosen according to the patients' actual conditions and exercise habits. The patients could do the simple housework, such as washing clothes, sweeping the floor, and buying vegetables, and could also do the exercises consuming little physical power, such as walking and doing Tai Chi. (4) Exercise intensity and frequency: it was best to keep the exercise at moderate intensity, with 55%–75% of the maximum heart rate during exercise. The exercise was performed 3–4 times a week with 30 minutes for a time. (5) Exercise records: the medical staff guided the patients to record their daily exercise, including the exercise time, exercise mode, heart rate, and other related contents. The medical staff should regularly check the patients' records, ask them about the problems of the exercise, and point out their mistakes to help them correct in time so as to ensure the correctness of the exercise. The patients were encouraged to ask questions to the medical staff, and the medical staff should give detailed answers to the questions to eliminate the patients' doubts and improve their treatment compliance. Both groups continuously received 6-week training.

### 2.4. Observational Indexes

(1) The patients' general data, including the sex, age, pathological type, pathological stage, smoking history, and education level, were compared. (2) The Piper Fatigue Scale (PFS) was adopted to evaluate the patients' cancer-related fatigue. This scale included four dimensions of affective meaning, behavior/severity, cognitive/mood, sensory, with 27 items in total. The total score of each item was 10 points, with 0 point representing none of fatigue, 1–3 points symbolizing mild fatigue, 4–6 points symbolizing moderate fatigue, and 7–10 points symbolizing severe fatigue. Total point = the sum of the score of every dimension/total number of the items. The Cronbach's *α* of PFS in this study was 0.89. (3) The 4-grade scoring method with 1–4 points was adopted to score the patients' pain, inappetence, insomnia and dyspnea, and higher scores indicated more severe symptoms. (4) The 6 minute walk test (6MWT) was adopted to measure the patients' walking distances within 6 minutes, and the operation method, matters needing attention and quality control of this test referred to the guidelines for 6MWT published by the American Thoracic Society (ATS) in 2002. (5) The patients' pulmonary function was compared between the two groups, and the evaluation indexes included the forced vital capacity (FVC), forced expiratory volume in 1s (FEV1), and FEV1/FVC% level. (6) The Quality of Life Questionnaire-Core Questionnaire (QLQ-C30) issued by the European Organization for Research and Treatment of Cancer (EORTC) was adopted to evaluate the patients' quality of life in the two groups, and this questionnaire included 30 items about walk, daily activities, adverse symptoms, mental status, and social support. Choosing “not at all,” “a little,” “quite a bit,” and “very much” will be scored one point, two points, three points, and four points, respectively, and higher scores represented worse quality of life.

### 2.5. Statistical Treatment

The statistical software SPSS20.0 was adopted for data processing and GraphPad Prism 7 (GraphPad Software, San Diego, USA) was used to draw graphs of the data in this study. The count data were tested by *x*^2^ and expressed by (*n* (%)). The measurement data were tested by *t* and expressed by ($\bar{x}$ ± *s*). When *P* < 0.05, the differences were considered statistically significant.

## 3. Results

### 3.1. Comparison of the General Data

No statistical difference in sex, age, pathological type, pathological stage, smoking history, education level, and other general data was observed between the two groups (*P* > 0.05; Table 1).

### 3.2. Comparison of the PFS Scores

Before intervention, no statistical difference in the affective meaning, behavior/severity, and cognitive/mood and sensory scores was observed between the two groups (*P* > 0.05). After intervention, the various indexes in the experiment group were lower compared with the control group (*P* < 0.05; Table 2).

### 3.3. Comparison of the Scores of Clinical Symptoms

Before intervention, no statistical difference in the scores of clinical symptoms, including the pain, inappetence, insomnia, and dyspnea, was observed between the two groups (*P* > 0.05). After intervention, the experiment group achieved eminently better improvement in clinical symptoms compared with the control group (*P* < 0.05; Table 3).

### 3.4. Comparison of the Walking Distances of 6MWT

Before intervention, no statistical difference in the walking distances of 6MWT was discovered between the two groups (*P* > 0.05). After intervention, the walking distances of 6MWT in both groups were increased, and the experiment group achieved observably longer walking distance compared with the control group (*P* < 0.05; Figure 1).

### 3.5. Comparison of the Patients' Pulmonary Function

Before intervention, no statistical difference in the various pulmonary function indexes in the two groups was discovered (*P* > 0.05). After intervention, the FVC, FEV1, and FEV1/FVC% level in the two groups were all improved, and the experiment group had signally higher indexes compared with the control group (*P* < 0.05; Table 4).

### 3.6. Comparison of the QLQ-C30 Scores

Before intervention, no statistical difference in the patients' QLQ-C30 score in the two groups was dicovered (*P* > 0.05). After intervention, the QLQ-C30 scores in both groups were decreased, and the experiment group achieved much lower score compared with the control group (*P* < 0.05; Figure 2).

## 4. Discussion

Lung cancer is a malignant tumor with a high incidence rate, and its incidence and mortality rates have shown a rising trend around the world. According to the statistical data [12], the incidence and mortality of lung cancer in males rank the first among malignant tumors, and its incidence in female ranks the third. As most patients have already suffered from medium and advanced lung cancer when they are diagnosed, they have such severe symptoms as cough, expectoration, fever, emaciation, cachexia, and dyspnea, which seriously threaten their daily activities and quality of life [13–15]. At present, the patients with medium and advanced lung cancer are mainly treated with radiochemotherapy, which can improve the patients' condition and increase their survival time. However, the radiochemotherapy may lead to such side effects as fatigue, weakness, pain, nausea, vomiting, and short breath during treatment, affecting the prognostic quality of life [16]. Hence, taking effective means to mitigate the clinical symptoms and enhancing the exercise capacity as well as quality of life is necessary. According to relevant studies [17], the training of aerobic function, with positive effects in improving the cardiopulmonary function and aerobic capacity, is an important method for rehabilitation treatment. In this study, the training of aerobic function was applied to the patients with medium and advanced lung cancer to improve their exercise endurance, clinical symptoms, and quality of life by doing certain amount of exercise at a certain speed and at a certain training intensity within a certain time.

The National Comprehensive Cancer Network (NCCN) recommends “exercise” as one of the most effective nondrug treatments for cancer-related fatigue [18]. This study assessed the patients' cancer-related fatigue with PFS and found that the affective meaning, behavior/severity, and cognitive/mood and sensory scores in the experiment group after intervention were lower compared with the control group (*P* < 0.05). This study result was in line with that of Ogawa et al. [19], suggesting that the training of aerobic function can mitigate the symptom of cancer-related fatigue in the patients with medium and advanced lung cancer. The reasons are analyzed as follows. The aerobic exercise enhances metabolism and reduces the patients' pain and limb stiffness and function decline caused by the reduced muscle strength level so as to accelerate the recovery of the physical efficiency. At the same time, the aerobic exercise can reduce the tension level of the patients' bodies and enhance their ability to regulate the internal and external environmental stimulation, lessening their stress level and relieving the fatigue. Besides, the patients' clinical symptoms were evaluated in this paper. Before intervention, no statistical difference in the scores of the pain, inappetence, insomnia, dyspnea, and other clinical symptoms was observed between the two groups (*P* > 0.05). After intervention, the experiment group achieved eminently better improvement in clinical symptoms compared with the control group (*P* < 0.05). After intervention, the FVC, FEV1, and FEV1/FVC% level in the two groups were all improved, and the experiment group had signally higher indexes compared with the control group (*P* < 0.05). According to the above results, the intervention effect of the training of aerobic function is significantly superior to the routine intervention measures. The training of aerobic function can mitigate such clinical symptoms as inappetence, insomnia, and dyspnea and improve the respiratory function. Besides, this training can decrease the oxygen consumption and blood viscosity and increase the ventilation function, vascular elasticity, cell viability, and oxygen uptake by improving the body's adaptability to upper limb motion. As a result, this training plays a role in the vasodilation, thus, improving the patients' pulmonary function and preventing the function decline [20–22]. The walking distance of 6 minute walk test (6MWT) is an important index to evaluate the patients' functional status and exercise endurance. In this study, the walking distances of 6MWT in both groups were increased after intervention, and the experiment group achieved observably longer walking distance compared with the control group (*P* < 0.05), indicating that the training of aerobic function can enhance the patients' exercise tolerance and its effect is eminently superior to the routine intervention measures. The training of aerobic function can promote the metabolism and prevent the function decline, rigid limbs, and pain caused by the reduced muscle strength level, ensuring the recovery of the patients' physical efficiency and enhancing their exercise endurance. In addition, this study evaluated their quality of life and found that the QLQ-C30 scores in both groups were enhanced after intervention, with the experiment group achieving much lower score compared with the control group (*P* < 0.05). These study results indicate that the training of aerobic function can mitigate such adverse symptoms as fatigue, pain, and dyspnea, improve their daily activity ability and pulmonary function, and ease the adverse emotions so as to increase their quality of life.

Aerobic exercise enhances the respiratory muscle strength, exercise capacity, and endurance through continuous strong stimulation, and its application effect is significantly superior to that of the simple conventional measures such as respiratory exercise and abdominal breathing [23–25]. Aerobic exercise can enhance the oxygen uptake capacity of skeletal muscles, stimulate the aerobic metabolism of local skeletal muscles, increase the endothelial surface area of the muscle capillaries, improve the efficiency of muscle mechanical contraction, and relieve the dyspnea occurred in the submaximal exercise. Therefore, the training of aerobic function, with significant effect on improving the pulmonary function and easing dyspnea, can increase the exercise endurance of the patients with medium and advanced lung cancer so as to speed up their recovery and improve living quality. The deficiencies of this study were as follows. The sample size was small, which might result in the deviation of the study results. The training methods of aerobic function were relatively single. Also, this study failed to conduct the follow-up to the patients. The subsequent studies should enlarge the sample size, enrich the training forms, further improve the experiment design, and conduct the follow-up so as to observe the long-term effects of the training of aerobic function on patients' clinical symptoms and quality of life.

In conclusion, the training of aerobic function has obvious therapeutic effect on medium and advanced lung cancer. This training can mitigate the cancer-related fatigue and clinical symptoms, improve the patients' pulmonary function, and enhance their athletic ability and quality of life. Therefore, this training possesses high application value in clinic.

## Figures and Tables

**Figure 1:** Comparison of the walking distances of 6MWT. The abscissa indicated before intervention and after intervention, and the ordinate indicated the walking distance of 6MWT (meters). The walking distance of 6MWT in the control group before and after intervention were (358.26 ± 45.23) and (392.19 ± 38.89), respectively. The walking distance of 6MWT in the experiment group before and after intervention were (352.49 ± 45.52) and (445.81 ± 35.05), respectively. ^*∗*^The remarkable difference in the walking distance of 6MWT between the two groups after intervention (*t* = 6.637, *P* < 0.001).

**Figure 2:** Comparison of the QLQ-C30 scores. The abscissa indicated before intervention and after intervention, and the ordinate indicated the QLQ-C30 score (points). The QLQ-C30 scores in the control group before and after intervention were (72.17 ± 5.53) and (56.36 ± 4.80), respectively. The QLQ-C30 scores in the experiment group before and after intervention were (73.05 ± 5.74) and (48.24 ± 4.03), respectively. ^*∗*^The remarkable difference in the QLQ-C30 score between the two groups after intervention (*t* = 8.396, *P* < 0.001).

**Table 1:** Comparison of the general data.

Observed indexes	Control group	Experiment group	*X* ^2^/*t*	*P* value
*Sex*				
Male	28 (66.67)	26 (61.90)	0.207	0.649
Female	14 (33.33)	16 (38.10)		
Mean age	58.31 ± 7.35	59.19 ± 7.63	0.538	0.592

*Pathological type*				
Adenocarcinoma	19 (45.24)	20 (47.62)	0.048	0.827
Squamous cell carcinoma	16 (38.10)	13 (30.95)	0.474	0.491
Small cell carcinoma	7 (16.67)	9 (21.43)	0.309	0.578

*Pathological stage*				
Stage III	30 (71.43)	32 (76.19)	0.246	0.620
Stage IV	12 (28.57)	10 (23.81)		
Smoking history	24 (57.14)	22 (52.38)	0.192	0.661

*Education level*				
College	13 (30.95)	15 (35.71)	0.214	0.643
Middle school	20 (47.62)	16 (38.10)	0.778	0.378
Primary school	9 (21.43)	11 (26.19)	0.263	0.608

**Table 2:** Comparison of the PFS scores.

Evaluation indexes		Control group	Experiment group	*t*	*P* value
Affective meaning	Before intervention	5.48 ± 1.29	5.55 ± 1.33	0.245	>0.05
	After intervention	4.55 ± 1.04	3.19 ± 0.86	6.531	<0.001
Behavior/severity	Before intervention	5.24 ± 1.45	5.43 ± 1.50	0.590	>0.05
	After intervention	3.95 ± 0.88	2.48 ± 0.67	8.613	<0.001
Cognitive/mood	Before intervention	4.88 ± 1.04	5.10 ± 1.16	0.915	>0.05
	After intervention	3.98 ± 0.92	2.83 ± 0.62	6.718	<0.001
Sensory	Before intervention	6.14 ± 1.35	6.07 ± 1.33	0.239	>0.05
	After intervention	4.29 ± 0.81	2.40 ± 0.73	11.233	<0.001

**Table 3:** Comparison of the scores of clinical symptoms.

Evaluation indexes		Control group	Experiment group	*t*	*P* value
Pain	Before intervention	3.05 ± 0.38	3.02 ± 0.47	0.322	>0.05
	After intervention	2.12 ± 0.33	1.86 ± 0.35	3.503	<0.001
Inappetence	Before intervention	3.38 ± 0.49	3.33 ± 0.48	0.472	>0.05
	After intervention	2.21 ± 0.56	1.76 ± 0.58	3.617	<0.001
Insomnia	Before intervention	3.36 ± 0.48	3.38 ± 0.49	0.189	>0.05
	After intervention	2.12 ± 0.49	1.69 ± 0.47	4.104	<0.001
Dyspnea	Before intervention	3.36 ± 0.53	3.33 ± 0.53	0.259	>0.05
	After intervention	2.48 ± 0.51	1.71 ± 0.46	7.266	<0.001

**Table 4:** Comparison of the patients' pulmonary function.

Evaluation indexes		Control group	Experiment group	*T*	*P* value
FVC (L)	Before intervention	2.36 ± 0.39	2.42 ± 0.41	0.687	>0.05
	After intervention	2.67 ± 0.58	2.98 ± 0.74	2.137	<0.05
FEV1 (L)	Before intervention	2.04 ± 0.43	2.10 ± 0.37	0.685	>0.05
	After intervention	2.55 ± 0.61	2.87 ± 0.53	2.566	<0.05
FEV1/FVC% (%)	Before intervention	62.70 ± 2.32	63.03 ± 2.47	0.631	>0.05
	After intervention	71.36 ± 3.16	79.19 ± 2.69	12.228	<0.05

## Data Availability

The data to support the findings of this study are available on reasonable request from the corresponding author.
